# Research and Simulation of Traditional Settlement Wind and Heat Environment Based on Computer Intelligent Computing Technology

**DOI:** 10.1155/2022/3715730

**Published:** 2022-07-21

**Authors:** Haoxi Chen, Xufu Zhang

**Affiliations:** ^1^Ph.D. Program in Cultural Heritage and Arts Innovation Studies, Taipei National University of the Arts, Taipei, Taiwan 11201, China; ^2^Department of Architecture, Kinmen National Quemoy University, Kinmen, Taiwan 89250, China

## Abstract

With the globalization of the world economy and the integration and heterogeneity of cultures, the collision between traditional settlements and local traditional culture, traditional culture and modern culture is gradually reduced. Traditional cultures, traditional settlements, and traditional architectural forms have gradually declined. Therefore, in the context of globalization, people are more concerned about how to recognize, understand, and inherit these traditions and traditional ways of life in the context of today's society and how to combine with the needs of contemporary communities to create an outdoor space suitable for human survival. However, due to the lack of research on traditional wind-heat conditions, there is no feasible evaluation method. Taking a typical village in Lianjiang County, Fuzhou as an example, various factors affecting wind-heat conditions in traditional villages are discussed in this paper. The CFD simulation technology is used to simulate and compare various types of settlements, and the wind and thermal environment around are compared and evaluated in detail and carried out in-depth research on it. By summarizing the general rules of natural ventilation of traditional residential buildings in Beigan Township, Lianjiang County, and Fuzhou, it is expected to be helpful to today's ecological construction. In order to construct a new type of energy-saving and land-saving community, some feasible methods and ideas are put forward to make it more realistic.

## 1. Introduction

German geographer Kohl discovered in the 1940s that communities are closely related to their surrounding geography and transportation. Since then, Jean Albert, an expert from Britain and France, has successively inspected the area and made a detailed division of the type and distribution of the area, thus forming the theoretical basis of the area [1]. Ronald in the United Kingdom was the first researcher to engage in rural architecture and villages. He believed that these villages were built by untrained amateurs, following local customs. Most of the materials selected came from local and only a few used foreign materials The material of the building and the function of the building has a crucial influence on the shape, and the aesthetics is often only ranked second [2]. These concepts embody the common denominator of communities around the world that have much less in common than the differences between them in terms of construction methods and construction ideas, and the current state of conservation is precarious and will continue. Therefore, the academic circles have carried out a detailed division of the villages and have begun to explore the local dwellings.

Although the concept of settlement is very broad from the beginning, from the existing research results, traditional villages, especially rural dwellings, have become a place of great research significance. With the deepening of people's understanding of the community, people's attention gradually shifted to the different forms of community and explored the origin and role of this difference [3]. Brian [4] believes that the main reasons for the differences are material and technological, environmental, social, cultural, political, economic, etc. Cardinale et al. [5] and Dili et al. [6] made an in-depth analysis of the formation and characteristics of British settlements from different perspectives, which are embodied in landscape environment, socio-economic, and political aspects. Dili et al. [7] pointed out that the traditional community refers to a specific social, political, and economic structure, which itself is a natural power. He analyzed large numbers of samples in order to look for differences in production to distinguish settlements. Since the last century, in-depth discussions on traditional villages in my country have been carried out and comprehensive results have been achieved in terms of content, method, breadth, and depth of understanding, etc.

Singh et al. [8] after visiting the local characteristic buildings in the European Mediterranean region, he felt that his house was in line with the living habits of the local residents. After testing the exterior and interior of the house, their exterior wall coverings got well. Although the temperature outside is constantly fluctuating, it has little impact on the interior, and the interior environment is more suitable for human life. Indraganti [9] in India investigated the living conditions of natives in hot, humid, and tropical monsoons. According to residents' opinions, residents generally feel that their residences are very comfortable, and the seasonal changes have not been greatly changed, which makes those living in modern times unable to adapt to this way of life. The reason for this is that when the Indians built their houses, they did not learn from ancient architectural styles or modern architectural styles, so when their houses were built, they did not consider modern architectural style, so their architectural style is not suitable for human life. From 1990 to 2000, the investigation of the wind-heat environment of local houses in China has not been deeply discussed [10]. Since this century, theories and methods about the wind-heat environment of traditional villages have been deepened, and the wind-heat problem has become a relatively independent research category, separated from the ecology of local architecture. Zhu and Liu sorted out the relationship between settlements and weather in Hubei and discussed the effect of traditional climate change [11]. Jiang [12] discussed the impact of climate change on the entire region of Hubei. Yang [13] discussed the role of ecological environment on community development from the perspective of sustainable development. After reviewing the relevant domestic and foreign literature, we believe that the existing research on the wind-heat environment of traditional settlements has made some progress, but compared with other related research results, it is insufficient [14–16].

The traditional wind-heat ecosystem has become a new subject, but the theoretical system, definitions, theories, basic scientific theories, and basic scientific methods are all ambiguous. So far, there is no theory or method on wind-heat problems. This makes the current research concept and research scope in this field unclear. From the perspective of community population, studies on wind-heat ecosystem are relatively rare. In addition, due to the characteristics of regional differences in research targets, there are also a considerable number of blanks in related studies in many places. Beigan Township, Lianjiang County, and Fuzhou traditional villages have yet to see the wind-heat ecological environment from the perspective of group living.

Taking a folk house in Beigan Township, Lianjiang County, and Fuzhou as an example, the wind-thermal environment of traditional villages in Beigan township, Lianjiang County, and Fuzhou was comprehensively analyzed by using computer numerical simulation technology. Based on the theory of numerical fluid dynamics, a numerical simulation of wind-thermal conditions in a representative village of Beigan Township, Lianjiang County, and Fuzhou was carried out. A new type of energy-saving and land-saving community is put forward to make it become a reality.

## 2. Analysis of Wind and Heat Environment of Traditional Settlements in Beigan Township and Lianjiang County

### 2.1. Analysis of Wind and Heat Environment in Beigan Township

Using computer intelligent numerical calculation technology, the distribution of temperature and wind speed flow field in Beigan Township is studied, and it is pointed out that the main factor affecting residents' living comfort is the temperature field 1.5 meters above the surface. Relative fluctuations in wind speed, temperature, etc.

### 2.2. Division of Beigan Township

The spatial structure and division of Beigan Township is shown in Figure 1. From the perspective of village texture, there are two different textures in the ancient village area of Beigan Township: one is the fine texture displayed by traditional villages and ancient streets and the other is the rough texture generated by the disorderly development of villages. In view of the wind and heat conditions of the village, according to the current situation of the ancient village in Beigan Township, the layout characteristics of its external space are divided into three regions A, B, and C, and the regional comparison is made. The indoor comfort, ventilation efficiency, and effectiveness of ventilation corridors were analyzed and evaluated.

The division from the densification mechanism of the partition can be divided into three partitions A, B, and C, each of which has different characteristics described in the division diagram shown in Figure 2.

1. Area A is a compact comb-like structure area, with Dashi Mountain on the west, Huangyang Mountain on the east, and Feng Shui Pond on the southwest. The overall street layout still maintains the dense “comb” layout of Beigan Township, thus forming a network structure of a village. This street is centered on South Gate Street, and the rest of the street runs inward along Main Street. The overall planning and layout not only reflects the ancient settlement's full respect for nature, but also is in line with the “feng shui” of Tibetan wind, qi, yin, and yang. It is the place where the descendants of the royal family of the Northern Song Dynasty lived.
2. Evolution pattern of regional B-type arrangement: in areas with complex terrain, with the continuous increase of population and scale of Beigan Township, a traditional village evolution mode characterized by a comb-like structure has gradually formed. Its characteristic is that the houses are arranged in a single form, the households are connected by inner lanes, and its transportation structure is also carried out according to its characteristics.
3. The C-shaped free-form building pattern mostly relies on the mountains and gradually rises according to the topography of the mountains, with scattered heights at the front and back. However, with the increase of the living population and the expansion of the living area, the existing comb-type community can no longer meet the living needs. Therefore, on the basis of the original comb-type community, a traditional comb-type community is formed, and under the local geographical features and convenient living conditions, according to the local characteristics, a residential area suitable for the living environment is designed.

### 2.3. Analysis of the Distribution of Wind and Heat Environment in Each District of Beigan Township

(1) A-type structure pattern in Beigan Township: area A is a relatively intact ancient village in Beigan Township and its distribution is characterized by dense, continuous, and small spacing. The house is located in the northeast, facing southeast, with dense buildings, mostly one-storey, with an average height of 4 meters, a lane width of 1.5 to 2 meters, and the height and width of the passage in the group is 2 to 3 meters. A narrow and dark passage was formed around it. The streets and alleys of the village are neat and orderly, forming an angle of 60 degrees with the main wind direction from the southeast. On the west side of the village, there is a large pond of about 200 meters, which constitutes the feng shui layout of “backward mountain and facing water.” Villages, buildings, and nature are integrated in a concentrated comb-like arrangement. On this map, each region has a color, one red, one blue, and one red dot, a number that represents a 1.75-degree Celsius rise.
  - Study on the simulation results of wind speed in the A zone
  - Figure 3 shows the distribution cloud of the wind field in Beigan Township. The southeast wind is the main wind direction. It can be seen from the flow velocity cloud map of the village that in the southeast of the mountainous area, due to the windy area, the wind force is very low, only 0.56∼1.40 m/seconds, and the flow rate is 3.1 m/s. Based on the geographical conditions of Beigan Township, we can conclude that the slope to the southeast of Beigan Township can prevent the summer monsoon in this area, because this area is not suitable for the high heat and high humidity monsoon in summer, so it should be properly blocked, even if it is different from the traditional site selection theory, it should be dealt with according to the specific environment, but it is also necessary to make reasonable adjustments to the traditional architectural experience theory, which is the architectural experience handed down from the local traditional settlements.
  - On the north side of block A, that is, on the leeward side, the wind speed is very low, and it is in a weak wind area below 1 m/s. The speed is about 1.1 m/s and the other areas are about 2.5 m/s. Overall, the air conditions in this area are good. In the streets, the maximum wind force is 0.8 m/s. In some areas, such as the outermost street entrances, such as in the southeast of the area, the speed can reach 2.5 m/s. Also, most of the area is in the dark blue class, with an average speed of less than 0.5 m/s, so the air circulation here is very weak. In general, the wind speed in the streets and lanes of Beigan Township A is about 1.0 m/s and about 2.5 m/s outdoors, which belongs to the appropriate speed range. Under the climatic conditions of summer in this area, the air velocity of open streets and alleys in most residential areas is 0.25∼1.4 m/s, which is within a safe range and suitable for living. However, in areas with high population density, the ventilation effect is generally poor, the wind speed in some areas is less than 0.25, which is not a suitable speed.
  - Study on the thermal simulation results of the A partition
  - Thermal radiation refers to the exchange of heat between the body and the surrounding air. Therefore, in order to feel comfortable in summer, there must be a good air circulation.  Figure 4 shows the temperature distribution cloud in area A of Beigan Township. The average temperature is 33.6 degrees Celsius. From the temperature changes in the village, it can be seen that the temperature in the area near the mountains and the two ponds is between 27.2 and 29.0 degrees Celsius. From a physical point of view, if the temperature drops by 1 degree Celsius, it is a kind of coolness. It can be seen from the above picture, since the west side is above the pool, the temperature will be below 30 degrees Celsius, so the climate in the western area is relatively better, while the temperature in the southern area has reached 39 degrees Celsius due to the relatively high density of buildings. The density of buildings in the central area and the narrow roads create a small heat accumulation area when the outdoor airflow is very low. The north-south direction of a street and lane of Nanmen Road in the area has maintained its original appearance. The height of the buildings on both sides of the street and lane has been increased and the road surface has been widened, that is, the overall dimensions of the block have changed. The direction of the incoming wind is at an angle of 15 degrees, between 37.7 and 39.5 degrees Celsius. Because the area is far away from the pond and affected by the high temperature, the overall thermal conditions of the entire area are relatively poor.
(2) The evolution pattern of B-type zoning structure: the new B-type community in Beigan Township is an evolution method arranged in a comb shape, which can be flexibly adjusted according to the actual local needs. The road layout of the new residential area in Zone B is fence-style, with the front facing south, forming an angle of 15 degrees with the main wind direction, and the two sides are parallel to the main wind direction of the incoming airflow. Compared with the conventional residential quarters, the height-to-width ratio of the new residential quarters has increased, and the height-to-width ratio of the new residential quarters is all on the second floor. According to the tunnel height of 6 meters and the width of the tunnel of 3 meters, the aspect ratio of the tunnel in the B area is 2, while in the conventional residential area, the aspect ratio of the tunnel is 2∼4, because only when the height and width are large, its occlusion effect will be better, and when the height and width of this area are smaller than that of conventional cells, the occlusion effect of this area will be significantly reduced.
  - Research on the simulation results of wind speed in B subarea
  - Beigan Township considers that the fluctuation of street wind speed in open residential structures outside the subarea is relatively stable, ranging from 0.28 to 1.4 m/s, which is a suitable value. From the data on Figure 5, the street wind speed in the subarea is 0.8 m/s. At the entrance of the tunnel downwind from the southeast, the wind speed at the entrance can generally reach 2.5 m/s because the wind direction is basically the same as the southeast monsoon wind direction. Indoors, the average wind speed in the leeward area is less than 0.8 m/s. Generally speaking, the average wind speed in area B is about 1.1 m/s, and the outdoor wind speed is about 2.2 m/s, which is in the appropriate wind speed range.
  - Analysis of thermal environment simulation results of partition B
  - Figure 6 is a cloud map of the temperature distribution in the southeast wind direction of subdistrict B in Beigan Township. The average temperature is 32.4°C. From the temperature cloud map of the settlement, the temperature near the mountain and two ponds is 29.0∼30.7°C. The incoming flow temperature is 31°C, which is nearly 1°C lower than the incoming flow temperature. From the cloud map of temperature distribution, it can be seen that the thermal environment in the western part of the subregion is still relatively good, because the blue low temperature area in the west is above the green water. Due to the concentration of buildings in the south and northeast areas of the subarea, the temperature is higher than that of the surrounding area. The temperature in the southern subarea is relatively high because the incoming wind from the building is blocked by the high ground. The roadway is wider than the original village. With very low outside wind speeds, this creates small areas of hot air accumulation.
(3) C-type building form of Block C in Beigan Township: block C in Beigan Township is built according to the mountains and does not need to be facing south. The building structure is relatively loose and the line of sight is relatively wide, usually with mountains as the background, facing the farmland. At the same time, restricted by topographical factors, the residential buildings are stacked layer by layer according to the natural slope of the hillside. Viewed from top to bottom, the distribution of buildings is highly scattered and evacuated at will, with a low-density living pattern.
  - Simulation study of wind field in area C
  - From the wind speed cloud in Figure 7 that the building arrangement along the east-west direction is beneficial to reduce air flow, but there is no such arrangement in the south and north regions, so it forms a strong contrast. In the northern part of the area, because of its high distribution density, the main airflow of the incoming flow is small, so the wind speed in the central area where the buildings in the northern part of the area are arranged is small, with an average speed of 0.5 m/s. However, because the southern part of the area is a belt-type evacuation structure, in order to facilitate air circulation, the wind speed at the entrance of this area is 2.2 m/s, the average wind speed in the road is about 0.8 m/s, and the wind speed at the end of the road reaches 1.1 m/s. The average wind speed is about 1.9 m/s, and the wind speed at the wind-guiding streets formed by this is significantly higher than the central building area with the density of the northern subdistrict. The results show that the air quality in the northern region is generally moderate, while the overall air quality in the southern region is good.
  - It can be seen from the wind speed cloud map that in the mountains near the north side of C, the average wind speed is only 0.8∼1.1 m/s and the minimum temperature in this area is 30.7 degrees Celsius. The wind does have a certain effect and is effective in heat insulation. In the case of using the peripheral-free arrangement, the area of the wind shadow area is relatively large, which makes the indoor air conditions of the peripheral arrangement relatively poor.
  - Simulation study of thermal conditions in area C
  - Figure 8 shows the temperature field in the southeast wind direction of the C area in Beigan Township. The average temperature is 32.4 degrees Celsius. According to the cloud map of the temperature distribution at point C in the settlement area, it is found that because the easternmost side is close to the pond, the temperature is low, forming a the relatively cold blue zone, with temperatures below 30 degrees Celsius. It can also be seen from the distribution curve of the temperature field that on the surface of the building and on the streets of the block, the higher the temperature range, the easier it is to appear on the surface of the building. The air temperature is lower in places closer to the sea. From the temperature of the clouds, different directions will also have different effects on the wind. The cluster structure in the south is dominated by east-west, while the community in the north is dominated by north-south, and its wind speed is significantly lower than that in the east-west direction, while it shows a better temperature distribution in the direction.

### 2.4. Evaluation of Comfort in Beigan Township

Through the analysis of the above simulation data in Beigan Township, the following results are obtained:

#### 2.4.1. The Overall Wind Condition of Beigan Township is Good

According to the wind direction, the wind environment of the three regions is analyzed. The results show: the best in the subregion B, the overall good in the subregion C, the subregion A is more sensitive than the subregion B and the subregion C. Comparison of wind and heat conditions in Beigan Township (see Table 1).

Assessment of comfort in each area of Beigan Township under wind conditions: Beigan Township is the hottest area in summer, and the average temperature in each area is above 25 degrees Celsius. According to this, the comfortable and uncomfortable speeds can be divided into different zones. The speed index is divided into various areas of Beigan Township and its suitable speed is carried out under the condition that the temperature is > 25 degrees Celsius and the wind speed is 0.7–2.9 m/s, as shown in Table 2.

### 2.5. Summary of Factors Affecting the Wind and Heat Environment in Beigan Township

This paper makes a detailed analysis and discussion of the wind and heat conditions of the settlements in Beigan Township from the whole to the local. It is believed that in order to adapt to and use nature, the ancestors adopted simple, concise, and economical methods. The settlement layout and many other factors create a comfortable living space. The overall wind temperature conditions in Beigan Township are very good. By comparing the wind temperature conditions in the three regions, the main wind directions of the three regions are obtained.

#### 2.5.1. The Location of the Village

Beigan Township is laid out according to the mountains and waters, and is built according to the mountains and in the villages. It can well reflect the local natural geographical environment and landform characteristics. This is because when Beigan Township is selected, it cleverly adopts the direction of southeast and northwest according to the characteristics of the terrain, instead of facing the south according to the traditional way. In addition, the slopes in the southeastern part of the area can better block the high temperature in summer, reduce the temperature of traditional settlements in Beigan Township, and create better microclimate conditions for the whole township, which is more conducive to the survival of residents.

#### 2.5.2. Spatial Structure

In order to ensure that the temperature in the micro-ring area will not be too high, the internal layout of the community becomes very critical, in which the streets and alleys are compactly arranged, the building groups are dense, the buildings are dense, and the mountain walls block the sunlight. The “high walls and narrow alleys” in Beigan Township are the characteristics of its traditional villages, which leads to the fact that most areas here are in a shady environment and there are many places that are not exposed to sunlight, so it can be very good here. Beigan Township is a new and old residential community. It is a brand-new and ancient community with a comb-like pattern as a whole. While most of them are in residential areas, and these alleys are ventilated, so the ventilation speed at the alleys of Beigan Township is relatively high, the wind speed in the alleys is relatively stable, and some areas are quiet areas. The roadways are shielded from each other, creating a cold surface on the ground, and with the open spaces such as courtyards and squares, a thermal pressure effect is generated, which provides better thermal pressure ventilation for the living area.

#### 2.5.3. Community Layout

The layout of the community is influenced by factors such as regional climate, geographic location, and the shape of its own buildings. In Beigan Township, under the sunlight in summer, the strong sunlight not only dazzles the villagers, but also increases the temperature. In the long-term living practice, the local people have accumulated a large number of architectural practices and adopted simple and economical construction methods to achieve this problem.

## 3. Conclusion

Taking a traditional village in Beigan Township, Lianjiang County, and Fuzhou as an example, the wind-thermal characteristics of traditional villages with different layouts were compared by using computer intelligent algorithm. Through summarizing and comparing the general rules of natural ventilation in Beigan Township, Lianjiang County, and Fuzhou, and analyzing them, some suggestions are put forward as a result.

1. Beigan Township, Lianjiang County, and Fuzhou is a representative traditional village. Its main wind and heat regime is dominant throughout the year and its main wind direction is summer. Under the condition of natural ventilation, Beigan Township, Lianjiang County, and Fuzhou generally adopts the layout of north-south or south-oriented, forming an Angle with the main wind direction to reduce incoming wind. When the included angle between the building layout and the air inlet is 0° to 90°, the wind speed in the outside wind area will decrease when the road entrance direction and the air inlet angle increase, and the wind speed will decrease when the angle increases.
2. By comparing the wind and heat conditions near the ground of residential areas under different layouts, the correlation between good ventilation and heating conditions and spatial layout is obtained, which lays a foundation for the design and evaluation of traditional residential building layout schemes. Beigan Township, Lianjiang County, and Fuzhou is a village with mountains and water on its back and good climatic conditions. The building space layout is clear, the space distribution is uniform, the space is continuous, and the building interval is short. Compared with the new living environment, the traditional residential area has the characteristics of high density and high plot ratio. In the winter climate of Fujian, the traditional comb layout and the entrance of roadway with large aspect ratio is an effective method.
3. The dense comb arrangement has better working conditions than the air condition, and the arrangement has the characteristics of dense, continuous, and small spacing. The high density building structure has poor natural ventilation capacity, resulting in the tail air intensity of the comb structure falling. But at the same time, it can effectively reduce the sunlight on the street, which is also good for the cooling of the building. The evolution patterns of the old and new hybrid layout patterns and comb structure patterns are carried out according to the two types of wind and heat. The lanes in the resettlement area are arranged in a grid pattern. The number of storeys and heights of homes built by new residents increased. It also increases the volume of traffic, improves the flow of traffic, improves the lighting, and increase the spacing between buildings but not conducive to the shielding between each other.

## Figures and Tables

**Figure 1:** Spatial structure and division of Beigan Township.

**Figure 2:** The densification mechanism of each partition.

**Figure 3:** Cloud map of SE wind direction and speed in Beigan township A.

**Figure 4:** Cloud map of SE wind direction and temperature distribution in subarea A.

**Figure 5:** Cloud map of SE wind direction and speed in subarea B.

**Figure 6:** Cloud map of SE temperature distribution in the dominant wind direction of partition B.

**Figure 7:** The wind speed cloud map of the dominant wind direction SE in partition C.

**Figure 8:** Temperature distribution map of SE in the dominant wind direction of partition C.

**Table 1:** Comparison of wind and heat environment in each zone.

	Section A	Section B	Section C
Comfort	Middle	Good	Optimal
The ventilation efficiency	Middle	Optimal	Good
Wind environment assessment	Middle	Optimal	Good

**Table 2:** Comparison of wind speeds in each zone.

Number	Model	Average wind speed (m/s)	Comfort evaluation
Section A	Intensive	0.563	Middle
Section B	Thin type	2.210	Optimal
Section C	Freestyle	1.324	Good

## Data Availability

The dataset used in this paper are available from the corresponding author upon request.
